The article "Lipoma of the Pancreas: A Rare Incidental Tumor" was retracted in 2024. Reasons: false authorship; unreliable results or conclusions; no approval from an author; concerns about the authorship.

# Lipoma of the Pancreas: A Rare Incidental Tumor

**DOI:** 10.7759/cureus.20122

**Published:** 2021-12-02

**Authors:** Mashhour F Alzarie, Abdullah A Alhaddab, Faris A Aljafar, Muhannad M Alzahrani, Doaa M Abdelaziz, Abdullah A Aleidan, Khalil I Alduraibi, Mohammed A Alfawaz, Mohammed T Khoja, Abdulwahab A Alshahrani, Hamad Y Alhassoun, Amal M Alshaibi, Abdullah A Alghizzi, Mazen D Aljohani, Faisal Al-Hawaj

**Affiliations:** 1 College of Medicine, King Saud University, Riyadh, SAU; 2 College of Medicine, Imam Abdulrahman Bin Faisal University, Dammam, SAU

**Keywords:** case report, computed tomography, incidental, pancreas, lipoma, abdominal pain

## Abstract

Recent studies have shown a significant increase in the utilization of computed tomography (CT) scans in the emergency department for a broad spectrum of conditions. This had a significant impact on the identification of patients with serious pathologies in a timely manner. However, the overutilization of computed tomography scans leads to increased identification of incidental findings. For example, pancreatic lesions are not uncommon findings that can be identified in imaging studies performed for other indications. Here, we report the case of a 55-year-old male with a history of urinary stone disease who presented with right flank pain and dysuria. The urinalysis findings revealed numerous red blood cells and leukocytes. Non-contrast computed tomography scan of the abdomen was performed to detect urinary stones, but no hyperdense stones were noted, suggesting the possibility of spontaneous passage of the stone. However, a lesion in the pancreatic tail was observed. This exhibited fat attenuation with no solid component in the pancreatic tail representing a pancreatic lipoma. No surgical intervention was made considering the benign nature of the incidentally detected tumor. Pancreatic lipoma is a very rare benign mesenchymal tumor of the pancreas. Recognition of the classic radiological feature of pancreatic lipoma is essential to avoid unnecessary investigation and procedures.

## Introduction

The use of cross-sectional images in the emergency department had increased significantly across a wide range of clinical presentations [1]. While imaging studies play a major role in the diagnostic process, their overutilization results in increased detection of incidental findings that can lead to unnecessary investigations and excessive referrals [2]. An incidental pancreatic lesion is an increasingly identified finding. For example, a retrospective study by Spinelli et al. that involved over 25,000 patients who underwent computed tomography (CT) scans of the abdomen revealed that the prevalence of incidental pancreatic cysts was approximately 1% [3]. However, not all pancreatic lesions are malignant and warrant surgical resection. Hence, careful clinical evaluation and accurate interpretation of such lesions are crucial to characterize these lesions to identify patients who require surgical intervention. It is generally suggested that pancreatic lesions measuring less than 2 cm are often benign [4]. Here, we report the case of a middle-aged male with renal colic who was found to have pancreatic lipoma, a very rare mesenchymal tumor of the pancreas.

The article "Lipoma of the Pancreas: A Rare Incidental Tumor" was retracted in 2024. Reasons: false authorship; unreliable results or conclusions; no approval from an author; concerns about the authorship.

## Case presentation

We present the case of a 55-year-old male who presented to the emergency department with a three-day history of right flank pain. The pain was radiating to his right groin. It was constant and stabbing in nature. He scored the pain as 8 out of 10 on the severity scale. It was exacerbated by passing urine and was partially relieved by over-the-counter analgesics. The pain was associated with nausea, vomiting, and difficulty in passing urine. There was no change in the urine color. The patient had a previous history of urinary stones, and he underwent lithotripsy three years ago. The patient is known to have hypertension, diabetes mellitus, and glucose-6-phosphate dehydrogenase deficiency. He did not undergo any previous surgeries. He was not known to have any food or drug allergies. He was a heavy smoker with 40 pack-years. He consumed alcohol occasionally. His family history was remarkable for inherited blood disorders, including beta-thalassemia and sickle cell disease.

Upon examination, the patient appeared in severe pain. His vital signs revealed tachycardia (122 bpm), normal respiratory rate (15 bpm), normal temperature (36.9°C), and maintained blood pressure (130/88 mmHg). He had normal oxygen saturation on room air. Abdominal examination revealed a soft and lax abdomen with no tenderness or palpable masses. Bowel sounds were of normal intensity and frequency. Examination of other systems revealed normal findings. Routine laboratory investigations did not reveal any abnormalities. Specifically, the urea and electrolyte levels were normal (Table 1).

**Table 1:** Summary of the results of the laboratory findings

Laboratory Investigation	Unit	Result	Reference Range
Hemoglobin	g/dL	14.5	13–18
Leukocytes	1000/mL	4.9	4–11
Platelet	1000/mL	380	140–450
Erythrocyte Sedimentation Rate	mm/hour	14	0–20
C-Reactive Protein	mg/dL	7.8	0.3–10
Total Bilirubin	mg/dL	0.5	0.2–1.2
Albumin	g/dL	3.9	3.4–5
Alkaline Phosphatase	U/L	50	46–116
Gamma-Glutamyltransferase	U/L	17	15–85
Alanine Transferase	U/L	16	14–63
Aspartate Transferase	U/L	18	15–37
Blood Urea Nitrogen	mg/dL	10	7–18
Creatinine	mg/dL	0.9	0.7–1.3
Sodium	mEq/L	139	136–145
Potassium	mEq/L	3.8	3.5–5.1
Chloride	mEq/L	104	98–107

Intravenous nonsteroidal anti-inflammatory drug (lornoxicam 8 mg) was administered to provide pain relief. The patient was asked to provide a urine sample for urinalysis. After the patient had provided the sample, he reported relief from his pain. The patient did not notice any stone while passing urine. The urinalysis findings had numerous red blood cells and leukocytes. However, the leukocyte esterase and nitrite were negative. Considering the aforementioned presentation, the initial diagnosis was a left-sided urinary stone that may have passed spontaneously. Subsequently, the patient underwent an unenhanced computed tomography scan of the kidneys, ureters, and bladder to detect any urinary stones. The scan did not demonstrate any evidence of hyperdense stones or hydronephrosis. However, a lesion in the pancreatic tail was noted. Hence, the scan was repeated with the administration of intravenous contrast. The scan revealed a non-enhancing, well-defined, lobulated lesion measuring 17 mm in the pancreatic head with fat attenuation (Figure 1). Such findings conferred the diagnosis of pancreatic lipoma. The patient was reassured that the lesion was completely benign and does not warrant any further investigation. However, considering the excessive anxiety of the patient about the lesion, the computed tomography scan was performed again after 12 months from the time of diagnosis. The scan demonstrated a stable appearance of the pancreatic lesion with no evidence of interval increase in its size or radiological features.

The article "Lipoma of the Pancreas: A Rare Incidental Tumor" was retracted in 2024. Reasons: false authorship; unreliable results or conclusions; no approval from an author; concerns about the authorship.

**Figure 1:** Axial (A) and coronal (B) abdominal CT images demonstrate a sharply demarcated lesion of fat density in the pancreatic tail (arrows) representing lipoma CT: computed tomography

## Discussion

We report an incidental finding of pancreatic lipoma in a middle-aged male with renal colic. Pancreatic lipoma is a type of pancreatic mesenchymal neoplasms, a group of tumors that arise from the non-epithelial structures of the pancreas, and they account for 1% of all pancreatic tumors [5]. Pancreatic lipoma was first described by Bigard et al. in 1989 as a hypoechoic pancreatic mass lesion on ultrasound examination [6], and the first computed tomography diagnosis of pancreatic lipoma was reported by Di Maggio et al. in 1996 [7]. Since the first reported case, the number of case reports of pancreatic lipoma does not exceed 200 cases [8].

Lipoma is a benign neoplasm composed of mature adipose cells within a collagenous capsule. Lipoma can develop almost in any region of the body [5]. The exact pathogenesis of lipoma remains unclear. It is proposed that diabetes mellitus, obesity, hypercholesterolemia, and family history may play a role. Further, the malignant transformation of lipoma into liposarcoma is uncertain [9].

The article "Lipoma of the Pancreas: A Rare Incidental Tumor" was retracted in 2024. Reasons: false authorship; unreliable results or conclusions; no approval from an author; concerns about the authorship.

A computed tomography scan can make the diagnosis accurately and preclude the need for biopsy and histopathological examination. As in the present case, the scan demonstrates a sharply demarcated homogeneous lesion of fat attenuation with no evidence of infiltration to adjacent structures [10]. However, the radiological differential diagnosis of lipoma includes liposarcoma, teratoma, and pancreatic lipomatosis. Focal fatty infiltration of the pancreas occurs with advanced age, metabolic syndrome, and certain inherited disorders such as cystic fibrosis [5].

Considering the rarity of the lesion, there are no established guidelines on the optimal management of lipoma. There are no definite criteria to distinguish between lipoma and liposarcoma. However, a small homogeneous lesion, measuring less than 3 cm in size, with no solid component can be diagnosed as pancreatic lipoma [10]. Pancreatic liposarcoma is extremely rare with limited radiological data available, but it tends to be larger in size. Magnetic resonance imaging can be helpful if there is any suspicion of the malignant behavior of the lipomatous lesion [11].

Since pancreatic lipoma is benign with virtually no risk of malignant transformation, surgical resection is not warranted. However, resection of the pancreatic lipoma may be required when the tumor is large and exerts a mass effect on vital structures or there is any suspicion for malignant transformation based on radiological features [8,9]. The concerning features include the presence of a solid mass in the lesion, thick septations, dilatation of the pancreatic ducts, and biliary obstructions [8].

## Conclusions

Pancreatic lipoma is a very rare benign mesenchymal tumor of the pancreas. A computed tomography scan can make the diagnosis accurately. This tumor is typically detected incidentally on cross-sectional images. Recognition of the classic radiological feature of pancreatic lipoma is essential to avoid unnecessary investigation and procedures. Since the tumor is completely benign, surgical resection is not advised in an asymptomatic patient with no suspicion of malignant transformation.
